The article "Long non‐coding RNA NORAD promotes the occurrence and development of non‐small cell lung cancer by adsorbing MiR‐656‐3p" was retracted in 2022. Reasons: manipulated images; unreliable data; unreliable results or conclusions.

# Long non‐coding RNA *NORAD* promotes the occurrence and development of non‐small cell lung cancer by adsorbing MiR‐656‐3p

**DOI:** 10.1002/mgg3.757

**Published:** 2019-06-17

**Authors:** Tianyu Chen, Shaoyun Qin, Yinan Gu, Huaqin Pan, Dachen Bian

**Affiliations:** ^1^ Department of Respiratory Medicine Jiangsu Taizhou People's Hospital Taizhou China

**Keywords:** *AKT1*, long non‐coding RNA, miR‐656‐3p, non‐small cell lung cancer, *NORAD*

## Abstract

**Background:**

To explore the role of non‐coding RNA activated by DNA damage (*NORAD*), a long non‐coding ribonucleic acid (lncRNA), in non‐small cell lung cancer (NSCLC) and its possible mechanism.

**Methods:**

Quantitative real‐time polymerase chain reaction was adopted for the detection of the expression levels of *NORAD*, micro RNA (miR)‐656‐3p, and AKT serine/threonine kinase 1 (*AKT1*). The effects of *NORAD*, miR‐656‐3p, and *AKT1* on cell proliferation and migration were examined through the Cell Counting Kit‐8 (CCK‐8) and Transwell assay. Subsequently, the binding relationships between miR‐656‐3p and *AKT1* and between miR‐656‐3p and *NORAD* were verified by dual‐luciferase reporter gene assay. Finally, the potential mechanisms of action of *NORAD* and miR‐656‐3p were explored through the torsion experiment.

**Results:**

The lncRNA *NORAD* expression level in NSCLC patients was notably higher than that in people in control group, that in patients with metastasis was higher than that in patients without metastasis, and that in patients with NSCLC in stage III‐IV was significantly higher than that in patients with NSCLC in stage I‐II. Elevation of *NORAD* stimulated the proliferation and migration of NSCLC A549/H460 cells. According to the reporter gene assay, *NORAD* could bind to miR‐656‐3p. Besides, miR‐656‐3p was significantly under‐expressed in cancer tissues of patients with NSCLC, and overexpression of miR‐656‐3p could block the proliferation and migration of A549/H460 cells and reversed promotion on cell proliferation and migration by *NORAD*. Furthermore, the reporter gene assay revealed that the overexpression of *AKT1*, a miR‐656‐3p target gene, could reverse miR‐656‐3p's inhibitory effect on the proliferation and migration of A549/H460 cells.

**Conclusion:**

LncRNA *NORAD* is capable of promoting the proliferation and migration of NSCLC cells, and its mechanism may be that it increases the *AKT1* expression by adsorbing miR‐656‐3p.

## 1 INTRODUCTION

Lung cancer is a malignant tumor, whose incidence and mortality rates were the highest worldwide, which seriously threatens human life and health (Jemal, Siegel, Xu, & Ward, 2010; McGuire, 2016; Wei, Tian, Song, Wu, & Liu, 2018). Based on pathological types, lung cancer can be divided into two types, namely, small cell lung cancer and non‐small cell lung cancer (NSCLC), and the incidence rate of the latter takes up 80%–90% of the total of lung cancer (Stewart et al., 2014). Currently, lung cancer is primarily diagnosed using imaging techniques. Although the growth and metastasis of NSCLC are relatively slow, most patients have been already in the middle and advanced stages when they are definitely diagnosed with the disease as there are no effective molecular markers for early diagnosis. At this time, cancer cells have undergone extensive invasion and metastasis, so the patients miss the best time for operation, which leads to the overall 5‐year survival rate of only about 17%. In terms of treatment, although there is an opportunity for early NSCLC to undergo surgical treatment, the radical cure rate is not high. Advanced NSCLC receives the comprehensive treatment dominated by chemotherapy, but the therapeutic effect is not satisfactory ("Cancer statistics", 2013). Therefore, lung cancer has become a major killer threatening human health. Investigating the mechanism of occurrence and development of lung cancer and finding molecular markers for early diagnosis of lung cancer are of great significance for early diagnosis and clinical treatment of lung cancer.

The article "Long non‐coding RNA NORAD promotes the occurrence and development of non‐small cell lung cancer by adsorbing MiR‐656‐3p" was retracted in 2022. Reasons: manipulated images; unreliable data; unreliable results or conclusions.

A long non‐coding ribonucleic acid (lncRNA) is a kind of linear RNA molecule which is abundant in various cells and has a length of more than 200 bases, but generally does not have the ability to code proteins (Chen et al., 2017). Current studies have manifested that varying lncRNAs can indirectly modulate the malignant behavior of cells, including malignant transformation, drug sensitivity, proliferation ability, and metastasis by participating in the regulation of various molecular mechanisms of malignant tumor cells (Gong et al., 2017; Zhang et al., 2016). However, more and more in‐depth studies have verified that lncRNAs also regulate the gene expression at both transcriptional and post‐transcriptional levels as well as the epigenetic level, so as to exert crucial effects on tumor initiation, progression, and metastasis, proving that they are potential prognostic markers and therapeutic targets for tumors (Hennessy, 2017; Shi et al., 2015). For instance, it has been demonstrated in some studies that lncRNA *UCA1* can regulate the proliferation of bladder cancer cells by acting on the *PI3K*‐*AKT*‐*mTOR* signaling pathway. Meanwhile, it has been confirmed that the transcription factor Ets‐2 can affect the expression level of *UCA1* and indirectly participate in the *AKT*‐mTOR signaling pathway to realize the regulation on cell apoptosis, thereby promoting the development of bladder tumor (Wu et al., 2013). Additionally, studies on lncRNA in lung cancer have been reported frequently. For instance, it has been found in some studies that *HOX* transcript antisense RNA (HOTAIR) exhibits a high expression in NSCLC tissues, and highly expressed HOTAIR often represents the poor prognosis of patients (Balci et al., 2016). According to other studies, lncRNA *KCNQ1OT1* located on human chromosome 11p15.5 has a close relationship to proliferation and drug resistance of lung cancer, and lowering its expression can remarkably enhance drug resistance of lung cancer to chemotherapeutic drugs (Du, Zhou, Beatty, Weksberg, & Sadowski, 2004; Ren, Xu, Huang, Zhao, & Shi, 2017). Moreover, it has been reported that lncRNA colon cancer associated transcript 1 (*CCAT1*) is primarily associated with malignant transformation of lung cancer, whose mechanism is probably to indirectly promote the c‐Myc activity in human bronchial epithelial cells induced by cigarette smoke exposure to induce malignant transformation, thereby promoting lung cancer's occurrence and development (Tran et al., 2015). However, the above research cannot explain all the phenomena, so it is very crucial to further study the effect of lncRNA on lung cancer.

The article "Long non‐coding RNA NORAD promotes the occurrence and development of non‐small cell lung cancer by adsorbing MiR‐656‐3p" was retracted in 2022. Reasons: manipulated images; unreliable data; unreliable results or conclusions.

It has been confirmed by existing studies that non‐coding RNA activated by DNA damage (*NORAD*), a lncRNA, plays a crucial role in varying tumors (Wang et al., 2018; Wu et al., 2017). In pancreatic cancer, for example, lncRNA *NORAD* can induce epithelial‐mesenchymal transformation caused by hypoxia to boost metastasis of pancreatic cancer (Li et al., 2017). Besides, in cervical cancer, *NORAD* is able to enhance the proliferation and invasion abilities of cancer cells by increasing the *SIP1* expression, so as to accelerate the process of tumors (Huo et al., 2018), but there is no research on the role of *NORAD* in NSCLC.

In this study, it was found that lncRNA *NORAD* exhibits an obvious high expression in NSCLC, so it was expected to further explore the role of *NORAD* in NSCLC and its potential mechanism.

## 2 MATERIALS AND METHODS

### 2.1 Ethical compliance

The research was approved by the Ethics Committee of Jiangsu Taizhou People's Hospital.

### 2.2 General data

Fresh NSCLC and NSCLC‐adjacent tissue samples of 24 NSCLC patients receiving surgical treatment were collected, and the NSCLC‐adjacent tissues should be at more than 5 cm from the edge of the tumor tissues. Besides, these patients had no history of other primary secondary tumors and no history of chemotherapy, radiotherapy, targeted therapy, etc. After collection, the samples were placed in a freezing storage tube, marked with sample information and stored in liquid nitrogen, and procedures in the whole storage and transportation process were operated under the condition with no enzyme. Meanwhile, clinicopathological data of all the patients were collected, including age, gender, smoking history, the tumor size, pathological subtypes, histological grades, TNM stages, and the lymph node status. All the patients voluntarily entered into this study and signed the written informed consent, and this study gained the approval of the Ethics Committee of the Jiangsu Taizhou People's Hospital.

The article "Long non‐coding RNA NORAD promotes the occurrence and development of non‐small cell lung cancer by adsorbing MiR‐656‐3p" was retracted in 2022. Reasons: manipulated images; unreliable data; unreliable results or conclusions.

### 2.3 Cell culture

HBE, a normal bronchial epithelial cell line, and SPC‐A1, H460, H1650, and A549, NSCLC cell lines, were all purchased from ATCC. The cells were cultured in Dulbecco's Modified Eagle's medium (Thermo Fisher Scientific, Waltham, MA) containing 10% fetal bovine serum (FBS; Hyclone, USA) or Roswell Park Memorial Institute 1,640 medium (GIBCO‐BRL; Thermo Fisher Scientific, Waltham, MA, USA) in a constant temperature incubator with 5% CO_2_ and saturated humidity at 37°C.

### 2.4 Cell transfection

At 1 day before transfection, an appropriate number of cells were seeded into six‐well plates and cultured in the cell culture medium without antibiotics, followed by transient transfection when the cells covered 60%–70% of the culture dish overnight. Then the cells were transfected with micro RNA (miR)‐656‐3p mimics, plasmid complementary deoxyribonucleic acid pcDNA‐*NORAD*, pcDNA‐*AKT1* and corresponding negative controls and mixed with Lipo2000. Subsequently, the mixture was let stand for 20 min after even mixing at room temperature to form the mimics/Lipo2000 (or DNA/Lipo2000) complex. Hundred microliters of the complex was slowly dripped into the culture solution and mixed well to co‐culture the cells for 4–6 hr. After that, the complex was removed, and the complete culture medium containing 10% FBS and 1% streptomycin was used to replace the culture medium for 24 hr for subsequent experiments. The siRNAs (si‐NC, si‐*NORAD*), miRNA mimics (miR‐NC, miR‐656‐3p), and overexpression plasmids (pcDNA‐NC, pcDNA‐*NORAD*, pcDNA‐*AKT1*) were synthesized by Shanghai GenePharma Co., Ltd. (Shanghai, China). They were cloned into the mammalian expression vector pcDNA3.1 (Invitrogen).

### 2.5 Total RNA extraction from tissues and cells

About 50 mg tissues were taken, ground in liquid nitrogen, and added with 1 ml TRIzol (Invitrogen, USA). Then cells were washed with PBS once after collection, added with 1 ml TRIzol at the cell density of 5 × 10^6^/ml. After that, the tissues or cells were fully homogenized, transferred to a 1. 5 ml centrifuge tube, and let stand for 5 min. Chloroform with a volume of 0.2 times that of the volume of TRIzol (1 ml TRIzol reagent needs 0.2 ml chloroform) was added into a centrifuge tube containing lysate, let stand for 5 min at room temperature after even mixing, and centrifuged for 10 min. Then the supernatant was transferred to another unused 1. 5 ml centrifuge tube, added with an equal volume of isopropyl alcohol, mixed evenly, and centrifuged for 10 min, and ultimately the supernatant was carefully sucked and discarded. After that, 1 ml of 75% ethanol was added into a centrifuge tube containing RNA precipitates, mixed uniformly, let stand for 5 min at room temperature, and centrifuged for 5 min. DNase 1 was applied to remove DNA in case of DNA contamination and the A260/A280 ratio was used to assess the quality of RNA. Finally, the supernatant was carefully sucked and discarded, and the RNA precipitates were dried at room temperature and dissolved in diethyl pyrocarbonate (DEPC)‐treated water according to their amount.

The article "Long non‐coding RNA NORAD promotes the occurrence and development of non‐small cell lung cancer by adsorbing MiR‐656‐3p" was retracted in 2022. Reasons: manipulated images; unreliable data; unreliable results or conclusions.

### 2.6 Quantitative real‐time polymerase chain reaction

After the concentration and purity of RNA samples were tested, cDNA samples were synthesized by reverse transcription with U6 and GAPDH as the internal reference, respectively. SYBR Green (Applied Biosystems, USA) premixed solution, templates, forward (F)/reverse (R) primers, and DEPC (Beyotime Biotechnology, China) were prepared into PCR solution, which was placed on a RT‐PCR instrument for PCR amplification. MiRNAs were reversely transcribed into cDNAs by miRNA RT Kit [Tiangen Biotech (Shanghai) Co., Ltd.], and PCR and quantitative analysis of miRNAs were carried out according to miRNA qPCR kit instructions [Tiangen Biotech (Shanghai) Co., Ltd.]. 2^‐△△ct^ method was applied to calculate the relative expression levels and the control genes were U6 and GAPDH. Primer sequences are listed below:

miR‐656‐3p (F: 5'ACACTCCAGCTGGGAATATTATACAGTCA 3',.

R: 5'CTCAACTGGTGTCGTGGAGTCGGCAATTCAGTTGAGAGAGGUUG 3');

U6 (F: CTCGCTTCGGCAGCAGCACATATA，R: AAATATGGAACGCTTCACGA);

*NORAD* (F: 5'TGATAGGATACATCTTGGACATGGA3'),

R: 5'AACCTAATGAACAAGTCCTGACATACA3');

GAPDH (F: 5'GAAGAGAGAGACCCTCACGCTG3', R: 5'ACTGTGAGGAGGGGAGATTCAGT3');

*AKT1* (F: 5'AGCGACGTGGCTATTGTGAAG3', R: 5'GCCATCATTCTTGAGGAGGAAGT3').

### 2.7 Luciferase enzyme detection

For the binding assay of miR‐656‐3p and *NORAD* or *AKT1*, complementary sequences for miR‐656‐3p and *NORAD* or *AKT1* predicted by bioinformatics analysis were synthesized chemically and inserted into the pGL3 vector carrying the Renilla luciferase (Rluc) gene to generate pGL3‐*NORAD* or pGL3‐*AKT1* for the luciferase reporter assay (the vectors synthesized by Shanghai GenePharma). The luciferase reporter plasmid or empty vector was co‐transfected into lung cancer cell lines with the encoding gene plasmid in a 24‐well plate. Luciferase activities were measured at 48 hr after transfection with the Dual‐Luciferase Reporter Assay System (Promega), according to the manufacturer's protocol. Rluc activity was normalized against firefly luciferase activity and presented as the percentage of inhibition.

The article "Long non‐coding RNA NORAD promotes the occurrence and development of non‐small cell lung cancer by adsorbing MiR‐656‐3p" was retracted in 2022. Reasons: manipulated images; unreliable data; unreliable results or conclusions.

### 2.8 Cell migration

A Transwell chamber was placed above a 24‐well plate. Then the transfected NSCLC cells were digested with trypsin and suspended in serum‐free medium, followed by counting with a cell counting plate. After that, the cells were diluted with serum‐free medium, whose density was adjusted to 1 × 10^5^/ml, and then the above cell suspension was added into the chamber. Then a culture medium containing 10% FBS was added into the sterile 24‐well plate for culture in an incubator. After 48 hr, the culture medium was removed, followed by washing with PBS, and the Transwell chamber was taken out and fixed with 4% paraformaldehyde for 30 min. After 0.5% crystal violet was applied for 10–15 min of staining, the staining agent was washed with PBS. Finally, observation and counting of the cells were performed using a microscope. All the experiments were repeated three times.

### 2.9 Cell proliferation

NSCLC cells after treatment were seeded into 96‐well plates at the density of 1 × 10^4^/well, followed by culturing for 0 hr, 24 hr, 48 hr, 72 hr, and 96 hr, respectively. Cell Counting Kit‐8 (CCK‐8) kit (Dojindo, Japan) was utilized to detect the cell proliferation ability, before which CCK‐8 and the culture medium were mixed at a ratio of 1:10 to prepare a mixed solution. The old culture medium was discarded, and 110 μl of the mixed culture medium was added for further 1 hr of incubation at 37°C away from light. Ultimately, the OD value at 450 nm was examined by enzyme‐linked immunosorbent assay, and six replicate wells were set in each group. All the experiments were repeated three times.

### 2.10 Western blotting

Cells were collected and lysed with RIPA lysis buffer (Beyotime, Beijing, China) with complete Protease Inhibitor Cocktail (Roche, USA). Equal amounts of protein lysates were subjected to 12% SDS‐PAGE gels and then transferred to PVDF membrane (Millipore, Billerica, MA). The membranes were incubated with the primary antibodies at 4°C overnight. The following primary antibodies were used: GAPDH (Cell Signaling, USA), *AKT1*(Cell Signaling, USA). After incubating with secondary horseradish peroxidase‐conjugated antibodies (Cell Signaling, USA) for 2 hr at room temperature, blots were visualized through an enhanced chemiluminescence system (Thermo Fisher Scientific, USA). Protein bands were quantified by densitometric analysis using Quantity One software (Bio‐Rad Laboratories, San Diego, CA).

The article "Long non‐coding RNA NORAD promotes the occurrence and development of non‐small cell lung cancer by adsorbing MiR‐656‐3p" was retracted in 2022. Reasons: manipulated images; unreliable data; unreliable results or conclusions.

### 2.11 Statistical methods

All data are presented as the mean ± standard deviation (*SD*) from three independent experiments. All statistical analyses were performed using SPSS 18.0 software (IBM, USA). Differences between groups were analyzed using Student's *t* test (two groups) or one‐way ANOVA analysis (multiple groups). A chi‐square test was applied to determine the association of *NORAD* levels with clinicopathological features. A value of *p* < 0.05 was considered statistically significant.

## 3 RESULTS

### 3.1 *NORAD* was obviously highly expressed in lung cancer and lung cancer cell lines

At first, the expression level of lncRNA *NORAD* in lung cancer tissues and corresponding cancer‐adjacent tissues was measured, and it was found that *NORAD* was obviously highly expressed in lung cancer tissues (Figure 1a). Second, lung cancer patients were divided into metastasis group and non‐metastasis group, and the expression level of *NORAD* in the two groups was examined. The results revealed that *NORAD* exhibited a notably high expression in the tissues of patients with cancer metastasis (Figure 1b). Thirdly, the expression of *NORAD* in different lung cancer stages were detected, which manifested that the expression of *NORAD* in patients with lung cancer in stage III–IV was markedly higher than that in patients with cancer in stage I–II (Figure 1c). Furthermore, the expression level of *NORAD* in lung cancer cell lines was also determined. According to the results, compared with that in HBE, the normal bronchial epithelial cell line, the *NORAD* expression level was generally high in lung cancer cell lines (Figure 1d). The above results indicate that *NORAD* may play a certain role in the process of lung cancer.

**Figure 1:** *NORAD* exhibits a remarkably high expression in lung cancer and lung cancer cell lines. (a) The expression of *NORAD* is obviously high in lung cancer tissues (*n* = 24) compared with that in cancer‐adjacent tissues (*n* = 24). (b) The *NORAD* expression in metastasis group (*n* = 16) is higher than that in non‐metastasis group (*n* = 8). (c) The expression of *NORAD* in the tissues of patients with lung cancer in stage III–IV (*n* = 18) is remarkably higher than that in patients with lung cancer in stage I–II (*n* = 6). (d) Compared with that in normal bronchial epithelial cells, the *NORAD* expression is generally high in lung cancer cell lines. *p < 0.05, **p < 0.01, ***p < 0.001

### 3.2 *NORAD* could evidently promote cell proliferation and migration

In order to explore the possible role of *NORAD* in lung cancer's occurrence and development, A549 and H460 cell lines were chosen for the following research. After transfection with *NORAD* overexpression plasmids, the *NORAD* expression in the two cell lines was evidently elevated compared with that in control group (Figure 2a). The effects of the *NORAD* expression on cell proliferation and migration were examined through the up‐regulation of its expression. The results denoted that the proliferation and migration of cells were markedly enhanced after the expression of *NORAD* was increased (Figure 2b–d).

The article "Long non‐coding RNA NORAD promotes the occurrence and development of non‐small cell lung cancer by adsorbing MiR‐656‐3p" was retracted in 2022. Reasons: manipulated images; unreliable data; unreliable results or conclusions.

**Figure 2:** *NORAD* can evidently promote cell proliferation and migration. (a) After lung cancer cell lines A549 and H460 are transfected with *NORAD* overexpression plasmids, the *NORAD* expression is markedly elevated. (b, c) Cell proliferation ability is obviously enhanced after the *NORAD* expression in A549 and H460 cells is upregulated. (d) Cell migration ability is remarkably improved after the *NORAD* expression in A549 and H460 cells is upregulated. *p < 0.05, **p < 0.01, ***p < 0.001

### 3.3 MiR‐656‐3p was a target gene of *NORAD*

It was found in bioinformatics analysis that miR‐656‐3p was a potential target gene for *NORAD*, and a potential binding site existed between the two (Figure 3a). Furthermore, the binding relationship between the two was verified through the dual‐luciferase reporter gene assay (Figure 3b,c). The expression of *NORAD* in A549/H460 cells was upregulated or downregulated to verify whether *NORAD* regulates the expression of miR‐656‐3p, and the expression level of miR‐656‐3p was detected. According to the results, the expression level of miR‐656‐3p was notably reduced after the expression of *NORAD* was upregulated, while it was increased after the expression of *NORAD* was downregulated (Figure 3d,e). Due to this regulatory relationship, the expression of miR‐656‐3p in lung cancer was further measured, which showed that miR‐656‐3P exhibited a significant low expression in lung cancer (Figure 3f).

**Figure 3:** MiR‐656‐3p is *NORAD*'s target gene. (a) Bioinformatics analysis shows that the two have potential binding sites. (b, c) Dual‐luciferase reporter gene displays that there is a binding relationship between them. (d, e) After the *NORAD* expression in A549/H460 cells is upregulated or downregulated, respectively, the miR‐656‐3p expression is notably decreased or increased. (f) Compared with that in cancer‐adjacent tissues (*n* = 24), miR‐656‐3p is significantly lowly expressed in lung cancer tissues(*n* = 24). *p < 0.05, **p < 0.01, ***p < 0.001

### 3.4 *NORAD* played its role by adsorbing miR‐656‐3p

Since *NORAD* could modulate the expression of miR‐656‐3p, it was speculated that *NORAD* lowered miR‐656‐3p to play its role. Then a torsion experiment was conducted to verify this speculation. In the first place, the transfection efficiency of miR‐656‐3p mimics was examined to ensure its effectiveness (Figure 4a). Then functional experiments denoted that upregulating the expression of miR‐656‐3p could markedly block the proliferation and migration of A549 and H460 cells, and can inhibited the promotion of *NORAD* on cell proliferation and migration in part (Figure 4b‐4e), which also confirmed the above speculation.

The article "Long non‐coding RNA NORAD promotes the occurrence and development of non‐small cell lung cancer by adsorbing MiR‐656‐3p" was retracted in 2022. Reasons: manipulated images; unreliable data; unreliable results or conclusions.

**Figure 4:** *NORAD* functions by adsorbing miR‐656‐3p. (a) The miR‐656‐3p expression is obviously upregulated after A549/H460 cells are transfected with miR‐656‐3p mimics. (b, c) The elevated miR‐656‐3p expression in A549/H460 cells can significantly inhibit cell proliferation and partially reverse *NORAD*'s promotion on cell proliferation. (d, e) The elevated miR‐656‐3p expression in A549/H460 cells can evidently suppress the cell migration ability and can partially reverse the promotion effect of *NORAD* on cell migration. *p < 0.05, **p < 0.01, ***p < 0.001

### 3.5 *AKT1* was a potential target gene of miR‐656‐3p

It was found in prediction and analysis through websites that *AKT1* was a potential target gene of miR‐656‐3p (Figure 5a), and the dual‐luciferase reporter gene assay further confirmed the binding relationship between the two (Figure 5b,c). The *AKT1* expression was measured after the expression of miR‐656‐3p was elevated in A549 and H460 cells, which displayed that both mRNA and protein expression levels of *AKT1* was remarkably inhibited (Figure 5d,e). We also found they have other binding sites, but the luciferase assay showed no significant difference (Supplementary Figure S1). The above results denote that *AKT1* is the target gene of miR‐656‐3p, and miR‐656‐3p can reduce the *AKT1* expression.

**Figure 5:** *AKT1* is a potential target gene of miR‐656‐3p. (a) Bioinformatics analysis manifests that the two have potential binding sites. (b, c) According to the dual‐luciferase reporter gene assay, there is a binding relationship between them. (d, e) After the expression of miR‐656‐3p in A549/H460 cells is upregulated, and the mRNA and protein expression levels of *AKT1* obviously declined. *p < 0.05, **p < 0.01, ***p < 0.001

### 3.6 MiR‐656‐3p exerted its effects by decreasing *AKT1*

Similarly, in order to explore whether miR‐656‐3p exerts its effects by decreasing *AKT1*, a torsion experiment was carried out. The experimental results confirmed that the proliferation and migration abilities of A549 and H460 cell lines were significantly enhanced after the *AKT1* expression was increased. However, the proliferation and migration abilities of cells were partially impeded after the expressions of both miR‐656‐3p and *AKT1* were upregulated compared with those after the elevation of the *AKT1* expression alone (Figure 6a,b), which indicates that miR‐656‐3p reduces the expression of *AKT1* to exert its effects. As *NORAD* was capable of downregulating the expression of miR‐656‐3p, the effect of *NORAD* on the *AKT1* expression level was expected to be verified. After the *NORAD* of expression was upregulated, it was found that *AKT1* was notably highly expressed at mRNA and protein levels compared with that in control group (Figure 6c,d), suggesting that *NORAD* upregulates the *AKT1* expression by adsorbing miR‐656‐3p.

The article "Long non‐coding RNA NORAD promotes the occurrence and development of non‐small cell lung cancer by adsorbing MiR‐656‐3p" was retracted in 2022. Reasons: manipulated images; unreliable data; unreliable results or conclusions.

**Figure 6:** MiR‐656‐3p exerts its effects by decreasing *AKT1*. (a, b) After the *AKT1* expression in A549/H460 cells rose up, the cell proliferation and migration abilities are notably enhanced, and miR‐656‐3p's inhibition on cell proliferation and migration are partially reversed. (c, d) After the *AKT1* expression in A549/H460 cells is upregulated, the mRNA and protein expression levels of *AKT1* are evidently increased. *p < 0.05, **p < 0.01, ***p < 0.001

## 4 DISCUSSION

As a class of highly conserved small non‐coding RNAs with 1825 nucleotides in length, miRNAs can suppress protein translation or degrade target genes at the post‐transcriptional level to regulate gene expression (Hayes & Chayama, 2016). It is well known that miRNAs play a role as oncogenes or tumor suppressor genes in the occurrence and development of cancer (Feng, Zhang, Wang, & Chen, 2015). In recent years, the competitive endogenous RNA (ceRNA) hypothesis has revealed a new mechanism of RNA interaction. In this case, non‐coding RNAs may act as competitive ceRNAs to play the sponge role of miRNAs, thus regulating the expression level of miRNA targets (Dawson, Harris, & Powell, 1990). Among them, the lncRNA, as a ceRNA, participates in the regulation of gene expression and varying biological processes, thereby promoting or inhibiting the occurrence and development of tumors, which is also relatively clear at present (Sterner, 1989; Zou et al., 2016). In prostate cancer, for example, lncRNA‐ROR can inhibit cell proliferation and invasion by adsorbing miR‐145 to upregulate the expression of downstream target genes (Liu et al., 2017). In breast cancer, lncRNA MIAT, as a ceRNA molecular sponge, competitively combines with miR‐155‐5p to achieve modulation of the expression of DUSP7 and promote the development of breast cancer (Luan et al., 2017). In lung cancer, it has also been reported that the lncRNA can be used as a ceRNA to modulate the expression of its target genes through interaction with miRNAs, thus participating in the development process of NSCLC (Li, Li, Yang, & Kang, 2018).

The article "Long non‐coding RNA NORAD promotes the occurrence and development of non‐small cell lung cancer by adsorbing MiR‐656‐3p" was retracted in 2022. Reasons: manipulated images; unreliable data; unreliable results or conclusions.

In this study, it was found that lncRNA *NORAD* was markedly highly expressed in NSCLC tissues and had a close relationship to tumor migration and staging. The expression of *NORAD* in A549 and H460, lung cancer cell lines, was elevated so as to further investigate the possible role of *NORAD* in lung cancer, and the CCK‐8 and Transwell assay were conducted to determine its effects on cell proliferation and migration. The results showed that *NORAD* significantly promoted cell proliferation and migration, suggesting that NORAD may be involved in the pathogenesis of lung cancer.

In order to further investigate the potential mechanism of action of *NORAD*, the bioinformatics analysis was performed, which revealed that miR‐656‐3p was its potential target gene. Additionally, it was confirmed by the dual‐luciferase reporter gene assay results that there was a binding relationship between the two, so it was speculated that *NORAD* also performed its role as a ceRNA. To verify this speculation, the expression of miR‐656‐3p in lung cancer was measured at first, which demonstrated that miR‐656‐3p exhibited an evident low expression in lung cancer tissues. After the *NORAD* expression was upregulated or downregulated, the expression of miR‐656‐3p was detected, and it was found that *NORAD* could notably modulate the expression of miR‐656‐3p. Subsequently, the expressions of miR‐656‐3p and *NORAD* in cells were simultaneously elevated. Functional experiments indicated that upregulating miR‐656‐3p could partially impede the promotion of *NORAD* on cell proliferation and migration, which also confirmed the abovementioned speculation.

In this study, it was confirmed that *AKT1* was the target gene of miR‐656‐3p, and miR‐656‐3p regulated the expression of *AKT1*, a member of the *AKT* (serine/threonine protein kinase) family (Weis & Hatton, 1989). At present, there are more and more studies revealing that *AKT1* plays a crucial role in tumors. For instance, in breast cancer and prostate cancer, the activation of *AKT1* can stimulate the proliferation of tumor cells, but at the same time it can suppress the migration ability of these cells (Gao, Alwhaibi, Artham, Verma, & Somanath, 2018; Riggio et al., 2017). This urges us to further explore what role *AKT1* plays in lung cancer. Torsion experiments denoted that elevating the *AKT1* expression could promote cell proliferation and migration and partially alleviate the miR‐656‐3p's inhibition on cell proliferation and migration, indicating that miR‐656‐3p may exert an effect by downregulating the *AKT1* expression. According to the speculation, *NORAD* upregulates the expression of downstream target genes by adsorbing miR‐656‐3p. For verification, the expression level of *AKT1* was examined after the *NORAD* expression in A549/H460 cells was upregulated. Based on the results, *AKT1* expression was markedly increased at the mRNA and protein levels, which also verifies the above speculation.

The article "Long non‐coding RNA NORAD promotes the occurrence and development of non‐small cell lung cancer by adsorbing MiR‐656‐3p" was retracted in 2022. Reasons: manipulated images; unreliable data; unreliable results or conclusions.

## 5 CONCLUSION

To sum up, it was found in this study that lncRNA *NORAD* could stimulate the proliferation and migration of NSCLC cells, and its mechanism was probably to adsorb and downregulate the miR‐656‐3p expression, thus upregulating the expression of *AKT1*, its downstream gene. This study not only provides a new idea for investigating the mechanism of NSCLC, but also provides a new perspective for its prevention and treatment.

## CONFLICT OF INTEREST

None declared.
